The article "Amorphous Selenium Nanoparticles Improve Vascular Function in Rats With Chronic Isocarbophos Poisoning via Inhibiting the Apoptosis of Vascular Endothelial Cells" was retracted in 2024. Reasons: unreliable data; unreliable results or conclusions; concerns about the images.

# Amorphous Selenium Nanoparticles Improve Vascular Function in Rats With Chronic Isocarbophos Poisoning via Inhibiting the Apoptosis of Vascular Endothelial Cells

**DOI:** 10.3389/fbioe.2021.673327

**Published:** 2021-06-24

**Authors:** Moli Zhu, Zhitao Gao, Yutian Fu, Yue Qiu, Keke Huang, Chaonan Zhu, Yinan Wu, Tiantian Zhu, Qianqian Wang, Lin Yang, Yaling Yin, Peng Li

**Affiliations:** ^1^School of Pharmacy, Xinxiang Medical University, Xinxiang, China; ^2^Collaborative Innovation Center of Henan Province for Green Manufacturing of Fine Chemicals, Key Laboratory of Green Chemical Media and Reactions, Ministry of Education, School of Chemistry and Chemical Engineering, Henan Normal University, Xinxiang, China; ^3^Chemistry and Chemical Engineering, Henan Normal University, Xinxiang, China; ^4^School of Laboratory Medicine, Xinxiang Medical University, Xinxiang, China; ^5^Department of Pharmacy, The First Affiliated Hospital of Xinxiang Medical University, Xinxiang, China; ^6^Basic Medical College, Xinxiang Medical University, Xinxiang, China; ^7^Sanquan Medical College, Xinxiang Medical University, Xinxiang, China

**Keywords:** amorphous selenium nanoparticles, isocarbophos, sodium hydrogen exchanger 1, apoptosis, human umbilical vein endothelial cells, vascular dysfunction

## Abstract

**Aim:**

This study aimed to investigate the preventive effect and possible mechanism of amorphous selenium nanoparticles (A-SeQDs) on isocarbophos induced vascular dysfunction.

**Methods:**

A-SeQDs was made by auto redox decomposition of selenosulfate precursor. Male rats were given isocarbophos (0.5 mg/kg/2 days) by intragastric administration for 16 weeks to induce vascular dysfunction. During the course, A-SeQDs (50 mg/kg/day) was added to the water from week 5. Then, the rats were killed to observe and test the influence of A-SeQDs on the vascular dysfunction induced by isocarbophos. Finally, human umbilical vein endothelial cells (HUVECs) were treated with 10% DMEM of isocarbophos (100 μM) for 5 days to detect the related indexes. Before the use of isocarbophos treatment, different drugs were given.

**Results:**

A-SeQDs could reduce total carbon dioxide, MDA, VCAM-1, ICAM-1, IL-1, and IL-6 while increasing oxygen saturation, NO content, and SOD activity in rats. A-SeQDs also resulted in relatively normal vascular morphology, and the expression of sodium hydrogen exchanger 1 (NHE1) and caspase-3 decreased in rats. Furthermore, in HUVECs treated with isocarbophos, A-SeQDs maintained mitochondrial membrane potential, inhibited the cleaved caspase-3 expression, and released cytochrome c from mitochondria to cytosol.

**Conclusion:**

A-SeQDs can inhibit the apoptosis of HUVECs through the mitochondrial pathway, and effectively treat the impairment of vascular endothelial function caused by isocarbophos, which is NHE1-dependent.

The article "Amorphous Selenium Nanoparticles Improve Vascular Function in Rats With Chronic Isocarbophos Poisoning via Inhibiting the Apoptosis of Vascular Endothelial Cells" was retracted in 2024. Reasons: unreliable data; unreliable results or conclusions; concerns about the images.

## Introduction

Organophosphorus(OP) belongs to phosphates-containing compounds such as phosphates or thiophosphates, which is harmful to humans in two ways, acute poisoning and chronic poisoning. Acute poisoning means that the body is exposed to a high concentration of OP for a short time, which inhibits the activity of plasma cholinesterase (AChE), leading to the accumulation of ACh in the synaptic endings of cholinergic neurons and the occurrence of muscarin-like and nicotine-like symptoms. In severe cases, coma, respiratory failure, and even death may occur. Patients with acute poisoning may also suffer from limb numbness, unresponsiveness, and other neurological dysfunction (Jo et al., 2014). Chronic poisoning refers to the long-term and low-dose exposure to OP compounds such as a small amount of skin, mucous membrane contact, and respiratory tract inhalation (Tsatsakis et al., 2012). AChE activity is not inhibited, but it will cause vascular function damage and neurocognitive dysfunction. Unfortunately, there is no good treatment for vascular dysfunction and cognitive impairment caused by OP (Pamies et al., 2014).

Fakhri-Bafghi et al. (2016) have found selenium-based drugs have protective effects on the toxicity of three common OP compounds to human erythrocyte *in vitro*. In addition, Na_2_SeO_3_ combined with VitC can reduce the toxic damage of OP compounds to the human body, but the effect of using Na_2_SeO_3_ alone is not obvious (Milošević et al., 2018). Although selenium protein or selenides have intrinsic biological activities (Alim et al., 2019), their safe doses *in vivo* are small, and they are prone to toxicity, limiting the application of traditional seleno compounds (Watanabe et al., 2020). At present, although selenium-based nanomedicine is widely used in biomedicine (Guan et al., 2018), it has insufficient intrinsic biological activity or natural aggregation and needs multi-layer modification to reach the target (Prateeksha et al., 2017). Therefore, it is vital to explore a safe and effective form of selenium with strong natural aggregation to give full play to the therapeutic effect of selenium.

Our laboratory has found that amorphous selenium nanoparticles (A-SeQDs) have intrinsic solid biological activity and natural selection aggregation. Through endocytosis and exocytosis, A-SeQDs can be accumulated in HepG2 cells, which has a reasonable prospect of drug development and application (Wang et al., 2016). Our study also showed that A-SeQDs could effectively reduce the occurrence of atherosclerosis and plaque development in rats by inhibiting sodium hydrogen exchanger 1 (NHE1).

The article "Amorphous Selenium Nanoparticles Improve Vascular Function in Rats With Chronic Isocarbophos Poisoning via Inhibiting the Apoptosis of Vascular Endothelial Cells" was retracted in 2024. Reasons: unreliable data; unreliable results or conclusions; concerns about the images.

Isocarbophos belongs to organophosphorus (OP) compounds, widely used in agriculture to control pests of rice and cotton (Badawy, 2020). In this study, we observed that A-SeQDs could significantly improve the structural and functional damage of the posterior cerebral artery in rats caused by chronic isocarbophos poisoning. Furthermore, in terms of mechanism, A-SeQDs may inhibit the activity of NHE1 and decrease the apoptosis of vascular endothelial cells via the mitochondrial pathway (Zhu et al., 2019).

## Materials and Methods

### Preparations of A-SeQDs

As described previously, selenium powder was added to sodium sulfite aqueous solution, and then bovine serum albumin was added. After that, the reaction system (pH = 6) was incubated at 20°C for 12 h. Finally, the dispersion was centrifuged, washed, and freeze-dried (Wang et al., 2016).

### Characterization

The 3D peak separation of A-SeQDs was detected by X-ray photoelectron spectroscopy (XPS). The size and morphology of A-SeQDs with an accelerating voltage of 200 kV were characterized by high-resolution transmission electron microscopy (HRTEM, JEOL JEM-2100). X-ray diffraction (XRD) measurements were conducted on a Bruker D8&Advance X-ray powder diffractometer with graphite monochromatized Cu Kα (λ = 0.15406 nm).

### Materials and Animals

Isocarbophos (Cat, LS93564) was provided by Hubei Sanonda Co., Ltd., (China). LiCl (Cat, LS34457) was the NHE1 agonist and was provided by Hubei Sanonda Co., Ltd., (China). Primary antibodies against NHE1 from Santa Cruz Company. Cytochrome C ELISA (Human Cytochrome C ELISA Kit ab221832) was purchased from Abcam Company. Male Sprague-Dawley (SD) rats (4 weeks old, 80 ± 100 g) were given by the Experimental Animal Center of Henan Province, license number: SYXK-Yu-005-0012). All rats were kept separately in cages at room temperature of 18–22°C for 12 h of light/dark cycling and free access to food and water. According to the recommendations in the guidelines for the Care and Use of Laboratory Animals of the National Institutes of Health, the feeding environment was strictly controlled. The animal experiment program was reviewed and approved by the Animal Care and Use Committee of Xinxiang Medical University.

### *In vivo* Experimental Design

All rats were randomly divided into six groups of six animals. Group 1: Saline group; Group 2: A-SeQDs (50 mg/kg) (Zhu et al., 2019) group; Group 3: LiCl (1 mg/kg, LiCl can induce cytoplasmic alkalization and act as an inhibitor of NHE1) (Kobayashi et al., 2000) group; Group 4: Isocarbophos (0.5 mg/kg/2 days) (Li et al., 2016) group; Group 5: Isocarbophos (0.5 mg/kg/2 days) plus A-SeQDs (50 mg/kg) group; Group 6: Isocarbophos (0.5 mg/kg/2 days) plus A-SeQDs (50 mg/kg) plus LiCl (1 mg/kg) group. The procedures for animal experiments were shown in Figure 2A.

The article "Amorphous Selenium Nanoparticles Improve Vascular Function in Rats With Chronic Isocarbophos Poisoning via Inhibiting the Apoptosis of Vascular Endothelial Cells" was retracted in 2024. Reasons: unreliable data; unreliable results or conclusions; concerns about the images.

### Determinations of Blood Gas Analysis, Inflammatory Factors, and Oxidation Indexes

Blood gas analysis indicators were determined in Xinxiang Ya-Shi-Jie medical testing institute for testing. In addition, inflammatory factors and oxidation indexes were measured according to the instructions of the commercial kit.

### Fundus Photography

Fundus photography was used to observe the fundus of rats anesthetized with sodium pentobarbital (30 mg/kg, I.P.). The fundus camera (Optomed, VET2) was used to monitor and photograph the optic nerve fundus. The fundus photography was based on the posterior polar area of the optical disc and retina. Changes in arterioles could be observed by examining the ocular fundus (Mojana et al., 2010).

### Determinations of Endothelium-Dependent Relaxation (EDR)

After the animals were anesthetized, the posterior cerebral artery was separated by carefully removing the adherent perivascular tissue, cut into a ring (3–4 mm in length), and then installed in an organ chamber infused with modified Krebs buffer. The contractile response was induced by treatment with phenylephrine (PE 1 μM). As mentioned earlier, when the contraction was in a plateau, accumulative acetylcholine (ACh) was added to trigger EDR to observe the effects of different drugs on vascular tension (Xue et al., 2018; Lobov and Dvoretskii, 2019).

### Pathomorphological Observation

After anesthetizing the animals, the posterior cerebral arteries were obtained and embedded in paraffin. Then paraffin sections were prepared by dehydration, transparency, wax dipping, and embedding. After that, Hematoxylin-eosin (HE) staining was performed and observed under the light microscope (magnification, x200; CX21BIM-SET5; Olympus Corporation, Tokyo, Japan). At the same time, the tissue prepared for electron microscope observation was observed under the electron microscope (Olympus Corporation, Tokyo, Japan).

### Detections of NHE1 by Immunofluorescence (IFC)

The vascular tissue was washed with cold PBS and incubated with 10% formalin PBS for 10 min. Tissues were sealed with 5% BSA for 30 min, then incubated with primary antibody at room temperature for 1 h. After washing with PBS, the sample was incubated with the fluorescent conjugated secondary antibody for 45 min. The pictures were taken under the fluorescence microscope.

### Detections of Caspase-3 by Immunohistochemical (IHC)

As described previously with modifications, paraffin sections of cerebral arteries were made. The sections were dewaxed with xylene and dehydrated through graded alcohol. Antigen retrieval was performed by pressure cooking in 0.01 M citrate buffer for 20 min. And then, the sections were incubated in endogenous peroxidase (DAKO) and protein block buffer to block endogenous peroxidase activity. After, the sections were incubated with primary antibodies at 4°C overnight. Next, the slides were incubated with a horseradish peroxidase-labeled streptavidin solution for 20 min at room temperature. Sections were finally stained with 3,3-diaminobenzidine tetrahydrochloride (DAB) and counterstained with hematoxylin. After dehydration and sealing, they were observed under the microscope. Semiquantitative analysis of tissue immunoreactivity was done.

The article "Amorphous Selenium Nanoparticles Improve Vascular Function in Rats With Chronic Isocarbophos Poisoning via Inhibiting the Apoptosis of Vascular Endothelial Cells" was retracted in 2024. Reasons: unreliable data; unreliable results or conclusions; concerns about the images.

### Cell Cultures and Cell Models

HUVECs were grown in the endothelial cell culture medium (Clonetics Inc., Walkersville, MD) from an American-type collection center. The medium was supplemented with 5% FBS, penicillin (100 U/ml), and streptomycin (100 g/ml). In this experiment, the cells were between the third and eighth generations. All cells were incubated at 37°C, 5% CO_2_, and 95% air. HUVECs were transfected with NHE1 expression plasmid or vector. The cells were inoculated in a 96-well plastic plate at a density of 5,000 cells/well. Then, different drugs were administered before OP treatment. HUVECs were treated with 10% DMEM of OP (100 μM) for 5 days. This concentration was chosen for this study because this OP concentration has been reported in the blood of people who are frequently exposed to OP (Huen et al., 2012) and patients with OP poisoning (Eyer et al., 2009). This concentration is also the same as that used in previous studies (Liu et al., 2009; Bharate et al., 2010).

### Plasmids and Transfection

Human NHE1 cDNA was derived from Origene Technologies (Rockville, MD, United States) and inserted into the pcDNA3.1(+) vector. The plasmid was transfected into HUVECs using Lipofectamine 2000 (Invitrogen; Thermo Fisher Science). The gene expression was detected 48 h after transfection. In order to stabilize the expression of NHE1, the transfected cells were transfected with plasmid or empty vector expressing NHE1. After adding 600 μg/ml G418 (Sigma Aldrich), the cells were selected for 2 weeks (Zhu et al., 2019).

### MTT Assay

The exponentially growing cells were incubated in 96-well plates (5 × 10^3^ cells/well) for 12 h and molded as described above. The experiment ended after 48 h incubation at 37°C. OD absorption values were recorded at 570 nm.

### Measurement of Intracellular pH (pHi)

As mentioned earlier, pH-sensitive fluorescent dye BCECF was used to measure pHi in HUVECs (Zhu et al., 2019). Cells grown on 35 mm plates were loaded with five μm BCECF-AM in the medium for 10 min. The fluorescence intensity was measured at alternating excitation wavelengths of 440 nm (pH-insensitive) or 495 nm (pH-sensitive) using the xenon lamp light source, and pHi in the cells was recorded. On the 530 nanometers, a fluorescence system with photomultiplier-based (Georgia Instruments, PMT-4000) was measured in 5 s. At the end of each experiment, the cells were established with a series of potassium pHi buffer, exposing the cells to the fluorescence ratio of the number phi and 495/440, and exposing the cells to a buffer containing the pHi of a potassium-containing 1 μM nigericin.

The article "Amorphous Selenium Nanoparticles Improve Vascular Function in Rats With Chronic Isocarbophos Poisoning via Inhibiting the Apoptosis of Vascular Endothelial Cells" was retracted in 2024. Reasons: unreliable data; unreliable results or conclusions; concerns about the images.

### Measurement of NHE1 Activity

The NHE1 activity was analyzed according to the previous method (Wang et al., 2005). After the HUVECs were treated, the NHE1 activity was determined by using the NH_4_Cl pulse method to determine the initial rate of the pHi value recovery. Briefly, after 10 min of dating with BCECF, the 30 mM NH_4_Cl was added to the medium. It was incubated for 5 min and was rinsed with Na^+^-free buffer. The cells were loaded with acid, and the value was reduced. When joining 100 mM NaCl, the NHE1 pump out of cell H^+^ increased in the original 40 s. This initial rate (dpHi/dt) was thought to reflect the NHE1 activity.

### Measurement of Intracellular Ca^2+^ ([Ca^2+^]i) Concentration

According to the instructions contained, the concentration of (Ca^2+^)i was measured using Invitrogen’s fluo-4 NW Kit (Wang et al., 2015). In short, HUVECs were treated according to the instructions, the culture medium was taken out, washed once with HEPES buffer (pH = 7.4), and added with 1 ml HEPES buffer containing fluorescent dye. After incubation for 30 min, the fluorescence intensity was measured at the excitation/emission wavelength of 485/520 nm.

### Calpain Activity

The calpain activity can be determined by using the fluorescent peptide Suc-Leu-Leu-Val-Tyr-AMC (calbiochem) as the substrate with a bit of modification under the method mentioned above (Dong et al., 2006). Soon, the cells were cultured in the medium with different treatment methods in 24-well plates. After being washed twice with PBS, the fluorescent peptide was added to a final concentration of 80 μM on PBS. Immediately after the addition of calbiochem, the fluorescence was recorded at 2 min intervals for 20 min at excitation 360 ± 20 nm and emission 460 ± 20 nm using a Synergy HT Multi-Detection Microplate Reader (BIO-TEK Instruments Inc.). The initial rate of peptidyl-AMC hydrolysis was used as the velocity of enzyme activity.

### Apoptosis Analysis

Annexin V-FITC Kit (Merk Millipore, Billerica, MA, United States) was used to detect apoptosis. In conclusion, the cells were washed and incubated with annexin V-FITC and propidium iodide (PI) in the dark for 15 min. Then, the stained cells were analyzed by flow cytometry (BD Biosciences, Franklin L, NJ, United States).

The article "Amorphous Selenium Nanoparticles Improve Vascular Function in Rats With Chronic Isocarbophos Poisoning via Inhibiting the Apoptosis of Vascular Endothelial Cells" was retracted in 2024. Reasons: unreliable data; unreliable results or conclusions; concerns about the images.

### Measurement of Δψm

According to the manufacturer’s instructions, the JC-1 mitochondrial membrane potential detection kit (Invitrogen; Thermo Fisher Scientific, Inc.) was used to detect mitochondrial membrane potential (Δψm). In short, cells were stained with JC-1 at 37°C for 20 min and analyzed by flow cytometry. The loss of Δψm was reflected by the decrease of red to green fluorescence.

### Cytochrome C ELISA

HUVECs were directly collected after treatment with different drugs, and subcellular components were prepared using a cell separation kit (ABCAM, AB109719). The fractions were treated and analyzed as described in the kit instructions. The concentration of cytochrome C was repeated with three different dilution ratios of the samples, and the standard curve of cytochrome C was used for interpolation. Draw inner interpolation (mean ± SD, *n* = 6).

### Statistical Analysis

All results were expressed as mean ± SD. Before making statistical comparisons, the Kolmogorov-Smirnov test was used to test the normal distribution of the data to determine whether ANOVA was appropriate. Then ANOVA was used for statistical comparisons between the groups, followed by Bonferroni’s *post hoc* test. Finally, statistical analysis was performed using GraphPad Prism 7 Software (GraphPad Software, San Diego, CA, United States), and *P* < 0.05 was considered to indicate a statistically significant difference.

## Results

### Characterization of A-SeQDs

In the presence of bovine serum albumin (BSA), A-SeQDs can be generated by autoredox reaction of sodium selenosulfate by adjusting the synthesis conditions (concentration of BSA and resting temperature) (Wang et al., 2016).

The XPS results of A-SeQDs showed (Figure 1A) that the peak of Se 3D was 54.93 and 55.77 eV, indicating that the sample was composed of selenium. XRD results (Figure 1B) showed that A-SeQDs had no characteristic diffraction peak, which proved its amorphous properties. The size and morphology of A-SeQDs were characterized by HRTEM (Figure 1C). In addition, the presence of diffuse halo ring in the selective electron diffraction (SAED) pattern of A-SeQDs verified that A-SeQDs was an amorphous sample (Figure 1D).

**FIGURE 1:** Characterization of A-SeQDs. **(A)** XPS spectra for A-SeQDs Se 3D. **(B)** XRD patterns of A-SeQDs. **(C)** HRTEM images of A-SeQDs, Scale bar: 20 nm. **(D)** SAED patterns of A-SeQDs. **(E)** Potentials of A-SeQDs in DMEM.

The article "Amorphous Selenium Nanoparticles Improve Vascular Function in Rats With Chronic Isocarbophos Poisoning via Inhibiting the Apoptosis of Vascular Endothelial Cells" was retracted in 2024. Reasons: unreliable data; unreliable results or conclusions; concerns about the images.

The Zeta potential analysis results showed that the Zeta potential of A-SeQDs in DMEM solution was −20.0 (Figure 1E). These prove that A-SeQDs has good stability and negative charge in physiological conditions.

### A-SeQDs Decreased Total Carbon Dioxide (TCO_2_) and Increased Oxygen Saturation (SPO_2_) in Rats With Isocarbophos

The animal experiment protocol is shown in Figure 2A. The body in an acidic environment is prone to aggravate inflammatory damage and oxidative stress injury. NHE1 pumps H^+^ out of the cell and binds to carbonate, resulting in increased CO_2_ production (Eatwell et al., 2013). As shown in Figure 2B, isocarbophos decreased SPO_2_ while increased TCO_2_ in the plasma of rats. A-SeQDs eliminated these adverse effects of isocarbophos in rats. A-SeQDs reduced TCO_2_ and increased SPO_2_ in the plasma of rats, which was statistically different from that of rats given isocarbophos alone (*P* < 0.05).

**FIGURE 2:** **(A)** The experimental protocols in the model of endothelial dysfunction in rats treated with A-SeQDs, Isocarbophos, or LiCl. **(B)** A-SeQDs significantly decreased total carbon dioxide (TCO_2_) and increased the oxyhemoglobin saturation (SPO_2_H). **(C)** A-SeQDs decreased oxidative stress response in rats. **(D)** Analysis of plasma inflammatory factor data in rats. Data were expressed by mean ± SD. *n* = 6, *p < 0.05, ***p < 0.001. Isocarbophos + A-SeQDs group vs. isocarbophos group.

The data (Table 1) also showed that the actual bicarbonate (AB), standard bicarbonate (SB), extracellular residual base [BE (ecf)], and whole blood residual base [BE(B)] values in all groups were within the standard range compared with the saline group, with no difference between the groups (*P* > 0.05).

**TABLE 1:** Blood gas analysis of rat serum.

**Group**	**AB (mM)^a^**	**SB (mM)^b^**	**BE (ecf)(mM)^c^**	**BE (B) (mM)^d^**
Saline	25.94 ± 1.70	17.89 ± 1.66	−4.28 ± 1.34	−6.01 ± 0.90
A-SeQDs	20.75 ± 3.11	18.09 ± 1.17	−4.37 ± 0.90	−5.85 ± 0.79
LiCl	21.36 ± 2.60	18.23 ± 1.59	−3.49 ± 0.67	−5.45 ± 0.66
Isocarbophos	21.72 ± 3.98	17.45 ± 0.91	−4.35 ± 0.97	−6.49 ± 0.86
Isocarbophos + A-SeQDs	20.53 ± 1.29	17.42 ± 0.96	−3.73 ± 0.43	−5.70 ± 1.02
Isocarbophos + A-SeQDs + LiCl	21.63 ± 3.37	17.53 ± 1.26	−3.4 ± 0.32	−6.79 ± 0.66

*Results of blood gas analysis in rats. ^*a*^AB (mM): actual bicarbonate; ^*b*^SB (mM): standard bicarbonate; ^*c*^BE (ecf) (mM): excess alkaline extracellular fluid; ^*d*^BE (B) (mM): excess alkaline blood. Data were expressed by mean ± SD. n = 6, isocarbophos + A-SeQDs group vs. isocarbophos group.*

### A-SeQDs Reduced the Level of Oxidative Stress and Inflammatory Response in Rats With Isocarbophos

As shown in Figure 2C, MDA content increased (5.15 vs. 1.68 nM, *P* < 0.05), while SOD activity (24.9 vs. 56.2 mM, *P* < 0.05) and NO content (12.2 vs. 22.9 μM, *P* < 0.05) decreased in the rats treated with isocarbophos. A-SeQDs could inhibit the effect of isocarbophos, which reduced MDA content (2.06 vs. 5.15 nM, *P* < 0.05) in rats and increased SOD activity (56.9 vs. 24.9 mM, *P* < 0.05) and NO content (20.9 vs. 12.2 μM, *P* < 0.05). These data suggest that A-SeQDs can significantly improve the oxidative stress injury induced by isocarbophos.

The article "Amorphous Selenium Nanoparticles Improve Vascular Function in Rats With Chronic Isocarbophos Poisoning via Inhibiting the Apoptosis of Vascular Endothelial Cells" was retracted in 2024. Reasons: unreliable data; unreliable results or conclusions; concerns about the images.

As shown in Figure 2D, the contents of ICAM-1 (409.4 vs. 148 nmol/g. prot, *P* < 0.05), VCAM-1 (78.5 vs. 32.9 μmol/g. prot, *P* < 0.05), IL-1 (547.4 vs. 291.8 nmol/g. prot, *P* < 0.05) and IL-6 (86.8 vs. 59.9 nmol/g. prot, *P* < 0.05) increased in rats treated with isocarbophos. A-SeQDs could inhibit the action of isocarbophos, decrease the contents of ICAM-1 (279.5 vs. 409.4 nmol/g. prot, *P* < 0.05), VCAM-1 (35.75 vs. 78.5 μmol/g. prot, *P* < 0.05), IL-1 (298.2 vs. 547.4 nmol/g. prot, *P* < 0.05), and IL-6 (37.4 vs. 86.8 nmol/g. prot, *P* < 0.05). These data suggest that A-SeQDs can reduce the inflammation induced by isocarbophos (Pedersen and Cala, 2004).

### A-SeQDs Alleviated Retinal Artery Stenosis in Rats With Isocarbophos

The mean diameter of the retinal artery was measured by fundus photography, which can be used to evaluate the microvascular injury correctly. As shown in Figure 3A, the mean diameter of the retinal arteries decreased, and the walls of vessels became roughened in rats given isocarbophos. Conversely, mean retinal artery diameters and vascular smoothness were increased in rats given both A-SeQDs and isocarbophos (Figure 3B).

**FIGURE 3:** A-SeQDs alleviated retinal artery stenosis and improved vascular function. **(A,B)** Retinal fundus artery imaging in rats. **(C,D)** Changes in vascular function in rats. Data were expressed by mean ± SD. *n* = 6, ***p < 0.001, isocarbophos + A-SeQDs group vs. isocarbophos group.

### A-SeQDs Increased the Endothelium-Dependent Relaxation (EDR)

EDR directly reflects the function of vascular endothelial cells. Endothelial function was determined by measuring Ach-induced endothelium-dependent relaxation (Yin et al., 2017). The decrease of EDR is a marker of vascular endothelial dysfunction. As shown in Figures 3C,D, compared to the rats of the saline group, isocarbophos could induce endothelial dysfunction of posterior cerebral arteries in the rats of vitro. Notably, 50 mg/kg of A-SeQDs significantly reversed the acute endothelial injury caused by isocarbophos.

### A-SeQDs Improved the Morphological and Structural Damage of the Posterior Cerebral Artery in Rats With Isocarbophos

As shown in Figure 4, HE staining results showed that various pathological changes occurred in the posterior cerebral arteries of rats given isocarbophos, including degeneration of vascular endothelial cells, dysplasia of smooth muscle, and rupture of elastic membrane. However, vascular morphology was healthier in rats treated with both A-SeQDs and isocarbophos.

The article "Amorphous Selenium Nanoparticles Improve Vascular Function in Rats With Chronic Isocarbophos Poisoning via Inhibiting the Apoptosis of Vascular Endothelial Cells" was retracted in 2024. Reasons: unreliable data; unreliable results or conclusions; concerns about the images.

**FIGURE 4:** A-SeQDs improve morphological and structural damage of the posterior cerebral artery. Morphological changes of the posterior cerebral artery in rats (100×). Observation of vascular endothelium in the posterior cerebral artery by electron microscopy in rats (12,000×). Six rats in each group.

The electron microscopic results showed that a variety of lesions appeared in the vascular endothelial cells of the posterior cerebral artery of rats given isocarbophos, including increased heterochromatin, hypertrophy of Golgi apparatus, and mitochondrial damage. However, the morphology of vascular endothelial cells was expected, and the organelles were not damaged in the rats treated with both A-SeQDs and isocarbophos.

### A-SeQDs Decreased the Expression of NHE1 in Bilateral Posterior Cerebral Artery Endothelium of Rats With Isocarbophos

The content of NHE1 in the posterior cerebral artery of rats was analyzed by immunofluorescence and western blotting. As shown in Figure 5A, immunofluorescence results showed that isocarbophos increased the NHE1 expression in endothelial cells of rat posterior cerebral artery. However, A-SeQDs could inhibit the expression of NHE1 in endothelial cells. The results of western blotting and immunofluorescence analysis were consistent (Figure 5A).

**FIGURE 5:** **(A)** Immunofluorescence was used to detect the expression of NHE-1 (green) and α-SMA (red) in the vascular endothelium of rats. DAPI staining showed that the nucleus was blue (200×). **(B)** The expression level of caspase-3 in the rat posterior cerebral artery was determined by immunohistochemistry (400×). Data were expressed as means ± SD. Isocarbophos + A-SeQDs vs. isocarbophos. Six rats in each group.

### A-SeQDs Reduced the Apoptosis of Rat Vascular Tissue Cells Induced by Isocarbophos

Caspase-3 is the most crucial terminal shear enzyme during apoptosis and the critical component of the CTL cell killing mechanism. In order to explore the reasons for the improvement of vascular function after A-SeQDs inhibition of NHE1 on vascular endothelium, we used immunohistochemical technique to detect the expression of caspase-3 in vascular tissue of the posterior cerebral artery. The results showed that the caspase-3 protein expression was significantly increased in the isocarbophos group compared with the saline group (Figure 5B). Thus, A-SeQDs could reduce the caspase-3 protein expression. These results suggest that A-SeQDs can reduce the apoptosis of vascular tissue induced by isocarbophos and protect the vascular tissue of rats.

The article "Amorphous Selenium Nanoparticles Improve Vascular Function in Rats With Chronic Isocarbophos Poisoning via Inhibiting the Apoptosis of Vascular Endothelial Cells" was retracted in 2024. Reasons: unreliable data; unreliable results or conclusions; concerns about the images.

### LiCl Activation of NHE1 Eliminated the Effects of A-SeQDs on Vascular Endothelial Function in Rats With Isocarbophos

Our previous study found that A-SeQDs can prevent endothelial dysfunction in high-fat and high-sugar rats by inhibiting NHE1 and has various protective effects on the cardiovascular system (Zhu et al., 2019). Therefore, we hypothesized that A-SeQDs might ameliorate the vascular endothelial injury caused by isocarbophos by inhibiting NHE1. To verify this idea, we treated rats with LiCl, an NHE1 activator, to observe whether LiCl affects the effect of A-SeQDs on endothelial dysfunction. The results showed that LiCl combined with A-SeQDs could eliminate the multiple impacts of A-SeQDs on posterior cerebral artery injury (Figure 4), retinal artery stenosis (Figures 3A,B), and vasodilatory response (Figures 3C,D). Furthermore, LiCl combined with A-SeQDs treatment could also eliminate the expression of NHE1 (Figure 5A) and caspase-3 (Figure 5B) and reduce the apoptosis of cells in the vascular tissues. The results suggested that inhibition of NHE1 by A-SeQDs was necessary for the prevention and treatment of endothelial injury with chronic isocarbophos poisoning.

### A-SeQDs Inhibited NHE1 Activation, Reduced pHi, and Inactivated Ca^2+^/Calpain Signals in HUVECs Processed by Isocarbophos

LiCl not only affects NHE1 but also affects cell metabolism. Therefore, we did the following work to investigate further the mechanism by which A-SeQDs reduced the apoptosis of vascular endothelial cells caused by chronic isocarbophos poisoning (Dong et al., 2006). We studied the effects of A-SeQDs on NHE1 activity, pHi, Ca^2+^ concentration, and calpain activity in HUVECs treated by isocarbophos.

HUVECs were infected with a lentivirus expressing NHE1 shRNA/NHE1 cDNA, and NHE1 gene expression was down-regulated/up-regulated. Isocarbophos (100 μM) was given 5 days earlier and used to mirror the microenvironment of vascular endothelial cells with chronic OP poisoning. After 5 days of treatment with isocarbophos (100 μM) in HUVCEs, NHE1 was significantly activated (0.559 vs. 0.223 ΔpH/min, *P* < 0.05; Figure 6A), the intracellular environment was alkalized (7.89 vs. 7.39, *P* < 0.05; Figure 6B), Ca^2+^ was overloaded (1,351.3.1 vs. 100%, *P* < 0.05; Figure 6C), and calpain activity was increased (316.1 vs. 100%, *P* < 0.05; Figure 6D), and the cell viability was weakened (0.601 vs. 0.846, *P* < 0.05; Figure 6E). These effects of isocarbophos were reversed in HUVECs with both A-SeQDs therapy and down-regulation of NHE1 expression by NHE1 shRNA. A-SeQDs lost these effects after NHE1 cDNA up-regulated NHE1 gene expression.

The article "Amorphous Selenium Nanoparticles Improve Vascular Function in Rats With Chronic Isocarbophos Poisoning via Inhibiting the Apoptosis of Vascular Endothelial Cells" was retracted in 2024. Reasons: unreliable data; unreliable results or conclusions; concerns about the images.

**FIGURE 6:** A-SeQDs can increase HUVECs activity by inhibiting NHE1 activation induced by isocarbophos, reducing pHi, and decreasing [Ca^2+^]i and calpain activity. Cultured lentivirus transfected HUVECs were co-incubated with isocarbophos (100 μM) for 5 days in the presence of A-SeQDs. **(A)** NHE1 activity was determined by the NH_4_Cl pulse method. **(B)** pHi was determined by the BCECF fluorescence method. **(C)** Fluo-4 fluorescence was used to detect the concentration of [Ca^2+^]i. **(D)** The fluorogenic peptide determined calpain activity. **(E)** Cell viability by MTT. Data were expressed as means ± SD. **p < 0.01, isocarbophos + NHE1-cDNA + A-SeQDs vs. isocarbophos + vector + A-SeQDs. *n* = 6.

### A-SeQDs Inhibited the Apoptosis of HUVECs Treated by Isocarbophos Through the Mitochondrial Pathway, Which Was NHE1-Dependent

NHE1 activated the cytochrome c-caspase3 signaling pathway in a Ca^2^^+^—dependent manner during ischemia-reperfusion, and promoted cardiomyocyte apoptosis (Wang et al., 2016). Cao et al. (2021) suggest that the potential protective mechanism of NHE1 on myocardial cells was related to the inhibition of the opening of mitochondrial permeability transition pore, the reduction of myocardial cell apoptosis, and excessive autophagy.

We examined the effect of NHE1 overexpression on the apoptosis of HUVECs to investigate the mechanism of A-SeQDs inhibiting the apoptosis of HUVECs treated with isocarbophos. Annexin-V and PI double staining showed that the apoptosis rate of the NHE1-cDNA plus isocarbophos group was higher than that of the vector plus isocarbophos group (21.5 vs. 8.5%, *P* < 0.05; Figure 7A). Figure 7B showed that the A-SeQDs treatment group reduced cleaved caspase-3 (the active form of caspase-3) in HUVECs treated with isocarbophos compared to the vector plus isocarbophos group. These suggested that A-SeQDs can indeed reduce the apoptosis of isocarbophos treated HUVECs at the cellular level by inhibiting NHE1. We examined whether NHE1-mediated apoptosis of HUVECs involved activation of mitochondrial pathways in the following experiments. The JC-1 method was used to measure the change of δψm, and it was found that A-SeQDs could reduce the increase of δψm in HUVECs treated by isocarbophos (98 vs. 64%, *P* < 0.05; Figure 7C). After the overexpression of NHE1, the above effect of A-SeQDs disappeared (25.2 vs. 64%, *P* < 0.05; Figure 7C). We also examined the release of cytochrome c from mitochondria to the cytosol by ELISA. The results showed that A-SeQDs could reduce the release of cytochrome C in the cytosol (11.1 vs. 30.9 ng/ml, *P* < 0.05; Figure 7E) and increase the content of cytochrome C in mitochondria (322 vs. 223 ng/ml, *P* < 0.05; Figure 7D) of HUVECs treated by isocarbophos. In contrast, these changes disappeared completely when NHE1 of HUVECs was overexpressed.

The article "Amorphous Selenium Nanoparticles Improve Vascular Function in Rats With Chronic Isocarbophos Poisoning via Inhibiting the Apoptosis of Vascular Endothelial Cells" was retracted in 2024. Reasons: unreliable data; unreliable results or conclusions; concerns about the images.

**FIGURE 7:** Overexpression of NHE1 promotes apoptosis through the mitochondrial pathway. **(A)** Apoptosis of HUVECs transfected with NHE1-cDNA plasmid, or vector was analyzed by flow cytometry after Annexin-V/PI staining. **(B)** IHC assayed protein levels of cleaved caspase-3 in HUVECs. The images showed a folding change in cleaved caspase-3 levels. **(C)** JC-1 assay was used to determine the change of Δψm. The loss of Δψm is mainly reflected by the change of fluorescence from red to green. **(D,E)** ELISA analysis of cytochrome c in cytosol and mitochondria. Overexpression of NHE1 promotes the release of cytochrome C from mitochondria into the cytosol. Data were expressed as means ± SD, ***p < 0.001. Isocarbophos + NHE1-cDNA + A-SeQDs vs. isocarbophos + vector + A-SeQDs, *n* = 6.

## Discussion

Among many biological nanomaterials, selenium-based nanomaterials are a special kind because they contain selenium. Most of the selenium compounds currently used for various medical purposes are nano selenium or selenium-naphthalene (Dorokhin et al., 2009). Although most nano selenium has good intrinsic biological activity, its natural aggregation is not very good, and it is still difficult to play an influential role at low concentrations (Dorokhin et al., 2009; Gunti et al., 2019). At present, most nano selenium needs multi-layer modification to play the effect (Menon et al., 2018). Multi-layer modification of materials will increase the cost, size, and complexity of the synthesis process, reduce repeatability and biocompatibility, etc. The synthesis of A-SeQDs can be controlled in our laboratory. Moreover, the synthesis method is simple, with high repeatability and small size. It can be entered into target cells through simple endocytosis, which has a great application prospect. Therefore, this paper takes A-SeQDs as the entry point to study the application of biological nanomaterials in the biomedical field, which has important theoretical significance and practical application value.

Chronic OP poisoning is different from acute OP poisoning in that AChE activity is not inhibited. But it causes vascular function damage and neurocognitive dysfunction. After entering the body, OP is oxidized by the cytochrome P450 system in liver particles to generate more toxic paraoxon, which is hydrolyzed by paraoxonase1 (PON1) and excreted in the urine in the form of a free or binding state with glucuronic acid, sulfuric acid, etc. (Muñoz-Quezada et al., 2016). In addition, besides decomposing lactones, PON1 also has antioxidant and peroxidase-like functions (Sunay et al., 2015). Therefore, chronic exposure to OP leads to a significant decrease in plasma PON1 activity and concentration, which increases the oxidative stress response (Vanova et al., 2018).

The article "Amorphous Selenium Nanoparticles Improve Vascular Function in Rats With Chronic Isocarbophos Poisoning via Inhibiting the Apoptosis of Vascular Endothelial Cells" was retracted in 2024. Reasons: unreliable data; unreliable results or conclusions; concerns about the images.

Our study showed that A-SeQDs decreased TCO2 and increased SPO2 and significantly inhibited oxidative stress and inflammatory response in chronic isocarbophos poisoning rats. Endothelial dysfunction can lead to restenosis plaque or endothelial injury caused by atherosclerosis. The mean diameter of the retinal artery measured by fundus photography can evaluate the vascular injury correctly. Treatment with A-SeQDs increased mean retinal artery diameter and smoothness in rats with chronic isocarbophos poisoning. In addition, after A-SeQDs administration, AChEmax was increased, AChEC50 was decreased, endothelium-dependent diastolic response and vascular lesion were improved in rats.

NHE1 is widely expressed in the plasma membrane of mammalian cells. It regulates pH and Na^+^ concentration through the intracellular and extracellular exchange of H^+^ and Na^+^. Activation of NHE1 increases intracellular Na^+^ leading to Ca^2+^ overload, which is considered a key factor in diabetes complications (Doliba et al., 2018).

We speculated that OP decreased PON1 and increased oxidative stress response after entering the body in view of the above studies. NHE1 is activated, pumping out intracellular H^+^ and extracellular Na^+^ in the presence of oxidative stress. As a result, the accumulation of Na^+^ activated Na^+^/k^+^-ATPase. Meanwhile, the Na^+^/Ca^2+^ reverse transport mechanism of the cell membrane and Ca^2+^/Mg^2+^ dependent endonuclease could be activated, leading to intracellular Ca^2+^ overload (Curtis et al., 2015). As a result, the cytochrome C-caspase3 signaling pathway was activated, the mitochondrial membrane potential decreased, and endothelial cell apoptosis occurred. At the same time, Ca^2+^ overload in vascular endothelial cells induces a large number of glycation end products (Hanahisa and Yamaguchi, 1998), which leads to impaired vascular function, decreases vascular elasticity, blood flow, and blood oxygen supply capacity. A-SeQDs can effectively reduce oxidative stress response and inhibit the damage of vascular endothelial function in rats treated with isocarbophos. The mechanism is related to inhibiting the expression of NHE1 in vascular endothelial cells, inhibiting the apoptosis of the cytochrome C-caspase3 signaling pathway, maintaining mitochondrial membrane potential, and reducing the apoptosis of vascular endothelial cells. This point is the innovation of this paper.

The article "Amorphous Selenium Nanoparticles Improve Vascular Function in Rats With Chronic Isocarbophos Poisoning via Inhibiting the Apoptosis of Vascular Endothelial Cells" was retracted in 2024. Reasons: unreliable data; unreliable results or conclusions; concerns about the images.

However, the detailed mechanism still needs to be further explored, the application value of A-SeQDs needs to be further explored, and the role of NHE1 in vascular injury caused by cardiovascular diseases needs to be further studied.

## Data Availability Statement

The raw data supporting the conclusions of this article will be made available by the authors, without undue reservation.

## Ethics Statement

The animal study was reviewed and approved by the Ethics Committee of Xinxiang Medical University (Xinxiang, China).

## Author Contributions

MZ performed most experiments and wrote the manuscript. ZG, YF, YQ, KH, CZ, YW, TZ, and QW partially performed some experiments. LY, YY, and PL conceived the whole project and revised the manuscript. All authors contributed to the article and approved the submitted version.

## Conflict of Interest

The authors declare that the research was conducted in the absence of any commercial or financial relationships that could be construed as a potential conflict of interest.
